RETRACTED

# Identification of RPS7 as the Biomarker of Ferroptosis in Acute Kidney Injury

**DOI:** 10.1155/2022/3667339

**Published:** 2022-10-13

**Authors:** Hao Zhang, Xuemei Liu, Lizhi Zhou, Zebin Deng, Yinhuai Wang

**Affiliations:** ^1^Department of Urology, The Second Xiangya Hospital at Central South University, Changsha, Hunan 410011, China; ^2^Department of Functional Medicine, Hunan Provincial Maternal and Child Health Care Hospital, Changsha, Hunan, China

## Abstract

**Objective:**

This paper aims to explore novel ferroptosis-related biomarkers for acute kidney injury (AKI).

**Methods:**

Various bioinformatic methods, such as differential expression analysis, functional annotation analysis, machine learning, and chemical-gene network analysis, were used in this study. Furthermore, the expression and proferroptotic role of RPS7 were validated with further bioinformatics analysis and biochemical experiments.

**Results:**

GSE30718 dataset and GSE139061 dataset were used, and the differentially expressed genes (DEGs) were screened. The DEGs were overlapped with ferroptosis-related genes and genes associated with AKI, which led to the identification of four candidate genes. Machine learning and ROC curve analysis were conducted, and RPS7 and TRIB3 were selected for diagnostic model analysis and functional analysis. Finally, the upregulation of RSP7 in cisplatin-induced AKI was validated in cisplatin-induced AKI, and its proferroptotic role was confirmed in cisplatin-treated proximal tubular cells.

**Conclusion:**

Our results indicated that RPS7 might present as a novel ferroptosis-related biomarker for AKI, and it derived ferroptosis to accentuate cisplatin-induced AKI.

## 1. Introduction

Acute kidney injury (AKI) is characterized by a sudden decrease in renal functions, manifested by increased serum creatinine levels and decreased urine volume [1]. AKI is commonly observed in clinical practice, especially in patients in the intensive care unit [2]. The etiology of AKI is quite complicated, which incorporates ischemia-reperfusion injury, sepsis, cardiac surgery, and the medication of nephrotoxic drugs [3]. The molecular mechanisms of AKI have been investigated for decades, and various aspects of mechanisms have been reported in the occurrence of AKI. In clinical practice, the diagnosis of AKI relies on serum creatinine level and 24-hour urine output, which may cause a low earlier diagnosis rate [4]. The serum creatinine level usually takes 2-3 days to rise, and the volume of urine sometimes increases slightly in part of AKI patients [5, 6] In this regard, identification of the novel markers for AKI is essential.

Ferroptosis is a type of nonapoptotic cell death denominated by Dixon in 2012 [7]. Unlike apoptosis, the bioprocess of ferroptosis is absent of chromatin margination and caspase activation [8]. The reduction of mitochondria crista is commonly observed in cells undergoing ferroptosis [8]; however, no specific morphological alterations were reported. Mechanistically, the execution of ferroptosis relies on overwhelming lipid peroxidation, which can be generated via the iron-catalyzed Fenton reaction or the lipoxygenase pathway [9]. Noteworthily, lipoxygenases are a family of iron-containing oxidases, which further stress the role of iron in the pathogenesis of ferroptosis [10]. The process of ferroptosis can be accelerated by increased intracellular iron and ROS generation. The overwhelming lipid peroxidation is inclined to be detoxicated by the enzymatic activity of GPX4, leading to the termination of ferroptosis [9]. Recently, it was manifested that therapeutic medication targeting ferroptosis alleviated various types of AKI [10], but the modulation of ferroptosis in AKI has not been fully elucidated. Noteworthily, our previous publication indicated that the ferroptotic process was ignited in the very early stage of cisplatin-induced AKI [11], suggesting that ferroptosis-related proteins may serve as early diagnostic markers for AKI.

RETRACTED

In this study, several AKI-related datasets were incorporated for bioinformatics analysis to identify novel genes related to the pathogenesis of AKI. In addition, a ferroptosis-related gene set, acquired from FerrDb database and GeneCards database, was used to explore the relevance of the newly discovered genes with ferroptosis. Finally, cisplatin-induced AKI model was used, and the biochemical experiments indicated that RSP7 might present as a novel potential ferroptosis-related biomarker for the diagnosis and treatment of AKI.

## 2. Materials and Methods

### 2.1. Datasets and Gene Collections

Three AKI-related datasets, i.e., GSE30718, GSE139061, and GSE165100, were obtained from the GEO database. GSE30718 dataset contains the renal transcriptional expression profile (array) of 28 AKI patients and 11 control samples. GSE139061 dataset includes the high-throughput sequencing data of 9 AKI renal samples and 10 control samples (human). GSE165100 dataset incorporates the renal transcriptional expression profile (array) of 4 cisplatin-induced AKI mice and 4 control mice. Ferroptosis-associated genes were acquired from FerrDb database (http://www.zhounan.org/ferrdb/current/) and GeneCards database (https://www.genecards.org/), and 659 genes were selected after merging and deduplication of the two databases.

### 2.2. Screening of the Candidate Genes for Ferroptosis in AKI

Firstly, the differentially expressed genes (DEGs) were authenticated between AKI and control samples in GSE30718 dataset (Limma package, version 3.44.3, *p* < 0.05) [12, 13]. Subsequently, the DEGs in GSE139061 dataset was also uncovered sing the “limma” package based on *p* value <0.05. WGCNA was used to filter AKI-associated genes in GSE30718 dataset. The R package “WGCNA” (version 1.70-3) was implemented to generate a coexpression network [14]. AKI samples were considered as trait data for WGCNA analysis, and turquoise module genes were retrieved as the ones highly associated with AKI. Finally, Venn diagram was applied to obtain the intersection DEGs, turquoise module genes, and ferroptosis-associated genes, followed by the identification of four candidate genes for ferroptosis and AKI.

RETRACTED

### 2.3. Functional Annotation Analysis

R package “clusterProfiler” (version 4.0.2) [15] for Gene Ontology (GO) and Kyoto Encyclopedia of Genes and Genomes (KEGG) enrichment analysis was used in our studies. Noteworthily, GO was subdivided into cellular component (CC), molecular function (MF), and biological process (BP). *p* < 0.05 was considered significantly different.

### 2.4. Recognition of Ferroptosis-Associated Biomarkers in AKI

Two machine learning methods, i.e., least absolute shrinkage and selection operator (LASSO) [16] and random forest (RF) [17], were applied to screen for disease characteristic genes. LASSO logistic regression in the R software package “glmnet” (version 4.0-2) was used, and the strong relevant features were selected. The RF method was deployed to obtain the feature genes with 5-fold cross-validation. The overlapping genes certificated by LASSO and RF were defined as characteristic genes in AKI. ROC curves were generated by the “pROC” package (1.17.0.1). Genes with AUC values of the ROC curve greater than 0.7 in both GSE30718 and GSE139061 datasets were identified as the ferroptosis-associated biomarkers in AKI.

### 2.5. Gene Set Enrichment Analysis (GSEA) Based on a Signal Gene

The GO, KEGG, and Reactome gene sets were used as the reference gene sets, and the AKI samples in GSE30718 dataset were sorted according to the correlation coefficients between the expression of all genes and the expression of biomarkers. GSEA was executed using the R software “clusterProfiler” (version 4.0.2) package. Significance thresholds were |NES| > 1 and *p* value<0.05.

### 2.6. Establishment of Cisplatin-Induced AKI Model

For *in vitro* studies, BUMPT cells (a mouse proximal tubular cell line) were maintained in culture media with high glucose DMEM, 10% FBS, and antibiotics. Lentivirus (acquired from Vigene Biosciences) was used to interfere with the expression profile of RPS7 in BUMPT cells. The cells were treated with 20 *μ*M cisplatin for 16-24 hours to induce tubular injuries *in vitro*.

RETRACTED

For *in vivo* studies, ethical approval was acquired from the Animal Ethical and Welfare Committee of the Second Xiangya hospital at Central South University (Approval number: 2022705). 8-12 weeks male C57BL/6 J mice were divided into the control group and the AKI group (6 mice in each group). Mice in the AKI group received an intraperitoneal injection of 25 mg/kg cisplatin to induce tubular injuries, while PBS solution was applied to the control group. The kidneys and serum samples were harvested two days later for further investigation.

### 2.7. H&E Staining

Kidney tissues were embedded in paraffin wax, and 4-*μ*m paraffin sections were obtained. The sections were deparaffinized and rinsed. Then, they were sequentially stained with hematoxylin for 3 minutes and eosin for 30 seconds. Finally, the sections were evaluated by light microscopy.

### 2.8. Immunoblotting

Kidney tissues or BUMPT cells were lysed by RIPA buffer, and the protein concentration was qualified. 15-30 *μ*g protein samples were subjected to 10-12% SDS-PAGE gel, and the separated proteins were transferred to PVDG membranes (0.22 *μ*m). The membranes were blocked and sequentially incubated with primary antibody and secondary antibody before the evaluation by the ECL detector. The primary antibody used in our study includes anti-NCOA4 (Bethyl Laboratories, catalog A302-272A; 1 : 1000), anti-FTH1 (Cell Signaling Technology, catalog 3998S; 1 : 1000), anti-GPX4 (Abcam, catalog ab125066; 1 : 2000), anti-RPS7 (Proteintech, catalog 14491-1-AP; 1 : 2000), and anti-*β*-actin (Proteintech, catalog 66009-1-Ig; 1 : 5000).

### 2.9. qRT-PCR Analysis

Total mRNA in kidney tissues or BUMPT cells was extracted with TRIzol (Invitrogen, catalog 15-596-026). The mRNA was reverse-transcribed into cDNA with the PrimeScript™ RT reagent kit (Takara). Finally, the cDNA was subjected to an ABI PRISM 7900 Sequence Detector System (Applied Biosystems) with ChamQ™ Universal SYBR® qPCR Master Mix (Vazyme). The calculated values compared with *β*-actin were used for statistical analysis. The primers incorporated in our study were RPS7-F: TGCTCGAGCTGGAGATG AAC; RPS7-R: GCTGTCAGGGTACGGCTTC; TRIB3-F: AGCAACTGTGAGA GGACGAAG; TRIB3-R: TGGAATGGGTATCTGCCAGC.

### 2.10. Immunofluorescence Staining

4-*μ*m sections were deparaffinized and permeated before antigen retrieval. Subsequently, the sections were blocked and incubated with primary antibodies overnight. The sections were rinsed and incubated with secondary antibody for 1 hour. DAPI was used to stain the nuclei, and the sections were scanned by fluorescence microscopy. The primary antibodies used in our study were anti-Megalin (Abcam, catalog ab76969; 1 : 500) and anti-RPS7 (Proteintech, catalog 14491-1-AP; 1 : 500).

RETRACTED

### 2.11. Immunohistochemistry Staining

4-*μ*m paraffin sections were deparaffinized, permeated, rinsed, and antigen retrieved. Subsequently, the sections were suppressed by H2O2 and blocked by goat serum. After that, the sections were sequentially incubated with anti-RPS7 antibody (Proteintech, catalog 14491-1-AP; 1 : 500) and secondary antibody before the application of DAB solution. Finally, the sections were evaluated by light microscopy.

### 2.12. MTT Assay

The cellular survive rate was detected by MTT assay. Cells were seeded into 96-well plates for overnight attachment. Cisplatin was used to prime the cells, and MTT solution (1 mg/ml Thiazolyl Blue Tetrazolium Bromide) were added for 4 hours after the treatment. The solutions were removed, and 150 *μ*l DMSO was added into each well. Finally, the plates were detected by a microplate reader (495 nm).

### 2.13. Statistical Analysis

The diagnostic model for ferroptosis-associated biomarkers was developed using the “lrm” function in R. All analyses were conducted using the R programming language, and the data from different groups were compared by the Wilcoxon test or Students' *t*-test. If not specified above, *p* value less than 0.05 was considered statistically significant.

## 3. Results

### 3.1. Screening of AKI-Related Genes

The DEGs between AKI and control samples in GSE30718 and GSE139061 datasets were authenticated, respectively, to uncover the variably expressed genes in AKI. 2692 DEGs (AKI vs. control), including 1934 upregulated genes and 758 downregulated genes in the AKI samples, were identified in GSE30718 dataset (Figures 1(a) and 1(b)). Meanwhile, a grand total of 2215 DEGs (AKI vs. control), including 811 upregulated and 1404 downregulated genes in the AKI samples, were determined in the GSE139061 dataset (Figures 1(c) and 1(d)). WGCNA analysis was applied to the data of GSE30718 dataset. Firstly, no outlier samples were excluded by sample cluster analysis (Figure 1(e)). Six were chosen as the optimal soft threshold (*R*^2^ = 0.85) to ensure that the interactions between genes maximally conformed to the scale-free distribution (Figure 1(f)). Next, a total of 5 modules were developed based on a gene clustering tree and dynamic tree cutting algorithm (setting the minimum number of genes per gene module at 100) (Figures 1(g) and 1(h)). The correlations between modules and AKI disease were computed, and turquoise module genes with the highest correlation were selected (Figures 1(i) and 1(j)). Hence, the 4568 genes in the turquoise module were regarded as genes closely associated with AKI. The DEGs and turquoise module genes were collected for further analysis.

RETRACTED

### 3.2. Identification of Potential Ferroptosis-Related Biomarkers in AKI

In order to recognize ferroptosis-associated genes in AKI, 659 ferroptosis-related genes were selected from FerrDb database and GeneCards database, and they were overlapped with the DEGs and turquoise module genes. Four intersecting genes, i.e., NRAS, TRIB3, TPM1, and RPS7, were identified (Figures 2(a) and 2(b)). The expression of these four genes in GSE30718 and GSE139061 datasets was illustrated in the heat maps (Figures 2(c) and 2(d)). The role of these four genes was explored by functional enrichment analysis. 185 GO items (146 BP items, 22 CC items, and 17 MF items) and 35 KEGG pathways were derived. The top 10 GO items under each classification and the top 15 KEGG pathways were showcased in bar charts (Figures 2(e) and 2(f)). The results revealed that these genes were involved in protein ubiquitination-related biological processes, vascular-associated smooth muscle cell migration, cellular response to reactive oxygen species, VEGF signaling pathway, Fc epsilon RI signaling pathway, EGFR tyrosine kinase inhibitor resistance, B cell receptor signaling pathway, ErbB signaling pathway, and Gap junction. In addition, the interactions between the four proteins and 20 other proteins were illustrated by GeneMANIA, and their functions were also characterized (Figure 2(g)).

Machine learning analysis was applied to the four candidate genes to further confirm their relevance with ferroptosis in AKI. As shown in Figures 3(a) and 3(b), three genes (NRAS, TRIB3, and RPS7) were picked out by LASSO logistic regression when lambda.min was 0.0241. Meanwhile, the same three genes (NRAS, TRIB3, and RPS7) were selected by RF model when the predicting accuracy of disease samples and normal samples was 0.8 (Figure 3(c)). Hence, three overlapping genes (NRAS, TRIB3, and RPS7) were obtained by crossing the genes filtered by two machine learning methods (Figure 3(d)). Subsequently, the ROC curves of the three genes were mapped in GSE30718 and GSE139061 datasets. As indicated in Figures 3(e) and 3(f), the AUC values of TRIB3 and RPS7 exceeded 0.7, suggesting that their expression profile could effectively distinguish AKI samples from control samples. Taken together, we reckoned that RPS7 and TRIB3 are highly potential ferroptosis-related biomarkers in AKI.

### 3.3. The Diagnostic Model and Functional Analysis of RPS7 and TRIB3

To verify the diagnostic value of TRIB3 and RPS7 in AKI, PCA analysis was conducted. The analysis of GSE30718 and GSE139061 datasets revealed that AKI samples and normal samples were largely in two different regions based on the expression of TRIB3 and RPS7, indicative of their diagnostic potency (Figures 4(a) and 4(b)). Subsequently, a diagnostic nomogram model based on the two ferroptosis-associated biomarkers was developed, which can predict an individual's risk and probability of suffering from AKI based on their expression profile (Figure 4(c)). In addition, the corresponding calibration curves were plotted to assess the validity of the diagnostic model. Our data revealed that the gap between the predicted probability and the actual probability was puny, suggesting that the model was reliable in predicting the risk of AKI (Figure 4(d)).

RETRACTED

Single-gene GSEA was performed based on the correlation coefficient between the expression of all genes and the expression of each biomarker (RPS7 and TRIB3, respectively) as a ranking criterion. Top 10 items under each gene set were displayed in Figure 5. RPS7 was associated with Ribosome, Proteasome, PI3K-Akt signaling pathway, Cytokine-cytokine receptor interaction, Natural killer cell-mediated cytotoxicity, and Hippo signaling pathway. TRIB3 was relevant to RNA splicing, NF-*κ*B binding, T cell chemotaxis, positive regulation of T cell migration, B cell homeostasis, and cell death in response to oxidative stress.

### 3.4. The Expression Profile of Ferroptosis-Associated Biomarkers in AKI

The expressions of RPS7 and TRIB3 were explored in multiple ways. As illustrated in Figures 6(a) and 6(b), RPS7 and TRIB3 were upregulated in AKI samples, as compared to control samples in GSE30718 and GSE139061 datasets. Similarly, the expressions of RPS7 and TRIB3 were conceivably increased in AKI samples in GSE165100 dataset (mouse) (Figure 6(c)). The expression profiles of RPS7 and TRIB3 were also investigated in *in vivo* and *in vitro* studies. Our qRT-PCR data showed that the mRNA level of RPS7 was very high in renal tubules, while the expression of TRIB3 was quite limited (Figure 6(d)). In this regard, RPS7 was selected for further investigations. Immunofluorescence staining demonstrated that RPS7 was extensively expressed in renal proximal tubular cells (marked by megalin) (Figure 6(e)). Cisplatin was used to induce AKI in BUMPT cells and mice. Within expectation, the expression of RPS7 was conceivably increased in cisplatin-treated BUMPT cells and mice kidneys, as validated by qRT-PCR analysis, immunoblotting, and immunohistochemistry staining (Figures 6(g)–6(j)).

### 3.5. RPS7 Promoted Ferroptosis in Cisplatin-Treated BUMPT Cells

Lentivirus was used to intervene in the expression of RPS7 in BUMPT cells. The overexpression or knockdown of RPS7 in BUMPT cells was initially validated by qRT-PCR studies and immunoblot analysis (Figures 7(a), 7(b), 7(e), and 7(f)). Our previous publication revealed that ferroptosis is an integral process in cisplatin-induced AKI, and we proceeded to explore the regulation of ferroptosis by RPS7 in cisplatin-related nephropathy. MTT assay revealed that RPS7 overexpression accentuated, while its gene disruption attenuated, cisplatin-induced BUMPT cell death (Figures 7(c) and 7(d)). The expressions of three ferroptosis markers, i.e., FTH1, GPX4, and NCOA4, were detected by immunoblotting. With expectation, a simultaneous decrease of the three markers was observed in cisplatin-treated BUMPT cells, which was accelerated by RPS7 overexpression but decelerated by RPS7 knockdown (Figures 7(g) and 7(h)).

RETRACTED

## 4. Discussion

In this study, bioinformatics methods were employed to analyze the online AKI datasets and ferroptosis-related gene sets, which uncovered four candidate genes for ferroptosis in AKI. Further investigations with machine learning and ROC curve analysis revealed that TRIB3 and RPS7 might be the potential ferroptosis markers in AKI, and their diagnostic values and functions were preliminarily explored. Subsequently, the expression of TRIB3 and RPS7 was validated in AKI datasets and laboratory investigations, which revealed that RPS7 might present as the ideal ferroptosis marker for AKI. Finally, the regulatory role of RPS7 on the ferroptotic process was validated in cisplatin-induced AKI.

AKI is characterized by high morbidity and mortality, and its molecular mechanism has not been fully elucidated. Traditional diagnosis methods with serum creatinine levels and urine output failed to meet the demand for early diagnosis [2]. Thus, it is urgently needed to identify novel potential biomarkers for AKI to facilitate its diagnosis and treatment in clinical practice. Bioinformatics is an efficient way to screen new biomarkers for various diseases, and their molecular mechanism and potential clinic relevance can also be calculated with certain algorithms. Bioinformatics analysis has been extensively used in the realms of AKI, leading to the discovery of multiple proteins. Yun et al. used GEO datasets to identify three previously uncovered genes (VMP1, SLPI, and PTX3) in the pathogenesis of sepsis-induced AKI [18], which presented several potential targets for future investigations. In addition, the analysis of human RNA sequencing data of AKI revealed 1160 DEGs, and a novel gene, i.e., STUB1, was identified as the key modulator of cisplatin-induced AKI [19]. Herein, we analyzed two human AKI-related datasets, which led to the determination of 2692 and 2215 DEGs, respectively (Figure 1). In addition, 4568 genes in the turquoise module, selected by CANNA analysis, were used as genes highly associated with AKI (Figure 1). The above-mentioned genes were involved in further bioinformatic investigations to identify novel biomarkers for AKI.

RETRACTED

Ferroptosis, a newly recognized type of nonapoptotic cell death, was recently reported to be involved in the pathogenesis of various types of AKI [10]. The process of ferroptosis mainly incorporated three aspects of metabolism: iron metabolism, lipid metabolism, and amino acid metabolism [9]. The increased free ferrous iron level, generated in the aberrant iron metabolism, catalyzed excessive lipid peroxidation to execute the cells [20]. Noteworthily, the lethal lipid peroxidation can be detoxicated by GPX4 and GSH, a process closely modulated by amino acid metabolism [21]. It was previously demonstrated that therapeutic medication targeting ferroptosis alleviated ischemia-reperfusion injury-, folic acid-, and rhabdomyolysis-induced AKI [22–24], and our previous publication indicated that ferroptosis is operative in cisplatin-induced AKI [11]. Recently, bioinformatics was extensively used in the realms of ferroptotic investigation to recognize its new regulators. The bioinformatics analysis by Liu et al. revealed that the MAPK1-related mRNA-miRNA-lncRNA axis participated in the ferroptotic process in cerebral hemorrhage [25]. Besides, Xu et al. reported using bioinformatics to identify PTGS2 and SQLE as the new ferroptotic genes involved in the immunotherapy of pancreatic adenocarcinoma [26]. In AKI scenarios, previous publications with bioinformatics revealed that miR-3587 and NFE2L2 are involved in the ferroptosis process [27, 28]. In the present study, we acquired 659 ferroptosis-associated genes from the online database, and these genes were overlapped with the DEGs and turquoise module genes, leading to the discovery of four genes related to ferroptosis and AKI (Figure 2). Further investigations revealed that RPS7 and TRIB3 were ferroptosis-associated biomarkers for AKI, and their potential drugs were predicted (Figures 2–4).

RPS7, in its full name small ribosomal protein subunit 7, is an essential part of the small subunit of ribosomes, and it participates in the bioprocess of protein synthesis in normal states [29]. Previous publications revealed that RPS7 is involved in the progression of various malignancies, such as prostate cancer and lung cancer [29, 30], but its role in renal injuries and ferroptosis has not been investigated. TRIB3, in its full name tribbles pseudokinase 3, was reported to play a pivotal role in cellular stress response [31]. The role of TRIB3 has been investigated in the pathogenesis of proteinuria-mediated renal fibrosis and diabetic nephropathy [32, 33]. In this study, our qRT-PCR data revealed that RPS7 was highly expressed in renal tubules while the mRNA level of TRIB3 was much lower (Figure 6). Due to the lack of data on kidneys and its high renal expression, RPS7 was selected for further investigation. Our biochemistry experiments showed that RPS7 was obviously upregulated in cisplatin-induced AKI (Figure 6). In line with the laboratory investigation, the bioinformatics analysis also demonstrated that the upregulated RPS7 may present a potential marker for AKI (Figures 4 and 6). Finally, the modulation of ferroptosis by RPS7 was explored in cisplatin-treated AKI. Within expectation, RPS7 accelerated ferroptosis to promote cisplatin-induced BUMPT cell death (Figure 7). Taken together, these data identified a novel ferroptosis-related marker for AKI and presented a new therapeutic target for cisplatin-related nephropathy; however, its molecular machinery needs further investigation.

RETRACTED

## 5. Conclusion

In conclusion, multiple databases were incorporated for bioinformatics analysis in this study, and the results identified RPS7 as a newly recognized marker for AKI. Moreover, we found that RPS7 participated in the modulation of AKI by accelerating ferroptosis.

## Figures and Tables

**Figure 1:** Screening of genes associated with AKI. (a and b) The DEGs in GSE30718 dataset. (c and d) The DEGs in GSE139061 dataset. (e and j) WGCNA analysis of GSE30718 dataset.

**Figure 2:** Identification of ferroptosis-related candidate genes in AKI. (a and b) The overlap of the DEGs, turquoise module genes, and ferroptosis-associated genes. (c and d) The expression of NRAS, TRIB3, TPM1, and RPS7 in GSE30718 and GSE139061 datasets. (e and f) Functional analysis of NRAS, TRIB3, TPM1, and RPS7. (g) GeneMANIA analysis of NRAS, TRIB3, TPM1, and RPS7.

**Figure 3:** Machine learning of ferroptosis-related candidate genes. (a and b) The analysis of LASSO logistic regression. (c) The analysis of RF model. (d) Overlap of the two machine learning methods. (e and f) The ROC curve analysis of NRAS, TRIB3, and RPS7 in GSE30718 and GSE139061 datasets.

**Figure 4:** The diagnostic model of RPS7 and TRIB3 in AKI. (a and b) PCA analysis of RPS7 and TRIB3 in GSE30718 and GSE139061 datasets. (c) The diagnostic nomogram model of RPS7 and TRIB3. (d) The calibration curves of the diagnostic model.

**Figure 5:** Single-gene GSEA of RPS7 and TRIB3. (a–c) Functional analysis of RPS7 based on GO, KEGG, and Reactome gene sets. (d–f) Functional analysis of TRIB3 based on GO, KEGG, and Reactome gene sets.

RETRACTED

**Figure 6:** The upregulation of RPS7 and TRIB3 in AKI. (a–c) RPS7 and TRIB3 were upregulated in AKI sample in GSE30718, GSE139061, and GSE165100 datasets. (d) The relative repression of RPS7 and TRIB3 in mice kidneys. (e) Immunofluorescence staining of RPS7 and megalin. (f) H&E staining and immunohistochemistry staining (RPS7) of the renal sections. (g–h) qRT-PCR analysis of RPSP7 in cisplatin-treated BUMPT cells and kidneys. (i and j) Representative immunoblot analysis of RPS7. CON: control; WT: wide type; CP: cisplatin; scale bars: 100 *μ*m; data are presented as mean ± SD.

**Figure 7:** RPS7 promotes ferroptosis in cisplatin-treated BUMPT cells. (a and b) qRT-PCR confirmed the intervention of RPS7 gene in BUMPT cells. (c and d) MTT assay showed that RPS7 overexpression accentuated, while its gene disruption attenuated, cisplatin-induced BUMPT cell injuries. (e and f) Immunoblot analysis confirmed the intervention of RPS7 gene in BUMPT cells. (g and h) Immunoblot analysis revealed that RPS7 overexpression accelerated, while its gene disruption decelerated, the depletion of FTH1, GPX4, and NCOA4 in cisplatin-treated BUMPT cells. CP: cisplatin; Lv-NC: empty vector lentivirus for RPS7 overexpression; Lv-RPS7: overexpression of RPS7 by lentivirus; shNC: empty vector lentivirus for RPS7 knockdown; shRPS7: knockdown of RPS7 by lentivirus; data are presented as mean ± SD.

## Data Availability

The experimental data used to support the findings of this study are available from the author upon request. Publicly available datasets analyzed in this study can be found in online repositories. GSE30718, GSE139061, and GSE165100 datasets were available in the GEO database (https://www.ncbi.nlm.nih.gov/geo/), and ferroptosis genes can be obtained from the FerrDb (http://www.zhounan.org/ferrdb/current/) and GeneCards (https://www.genecards.org/) databases.
